The article "Nonenzymatic Glucose Sensor Based on Porous Co3O4 Nanoneedles" was published in 2022. Journal: J Environ Public Health.

# Nonenzymatic Glucose Sensor Based on Porous Co_3_O_4_ Nanoneedles

**DOI:** 10.1155/2022/6442241

**Published:** 2022-10-08

**Authors:** Jianchun Sun, Hongjing Zhao, Zhongchang Wang

**Affiliations:** ^1^College of Metallurgy and Materials Engineering, Chongqing University of Science and Technology, Chongqing 401331, China; ^2^Chongqing Ecological Environment Minitoring Center, Chongqing 400030, China; ^3^International Iberian Nanotechnology Laboratory, Braga 4715-330, Portugal

## Abstract

Herein, porous Co_3_O_4_ nanoneedle arrays were synthesized on nickel (Ni) foam (Co_3_O_4_ NNs/NF) by one-step hydrothermal method. Some electrochemical methods were used to investigate its nonenzymatic glucose sensing performance in alkaline solution. The results show that the sensitivity of Co_3_O_4_ NNs/NF electrode to glucose is 4570 *μ*A mM^−1^ cm^−2^. The linear range is 1 *μ*M-0.337 mM, and the detection limit is 0.91 *μ*M (*S*/*N* = 3). It also displays good selectivity and repeatability for glucose. The good electrochemical sensing performance of Co_3_O_4_ NNs/NF based sensor for glucose can be attributed to interconnected porous structure and large specific surface area of Co_3_O_4_.

## 1. Introduction

Rapid and accurate detection of blood glucose concentration is very important for the diagnosis and treatment of diabetes. Although graphene oxide based glucose sensor dominates the market, it has some defects, such as high cost, limited stability, and complex enzyme immobilization process [1, 2]. In recent years, nonenzymatic glucose sensors have attracted the attention of a large number of researchers because of their advantages such as low cost, good stability, fast response, and simple fabrication [3].

Electrocatalytic active materials modified on the electrode surface have a great impact on the performance of nonenzymatic glucose sensor [4]. So far, a series of nanostructured materials based on precious metals and their alloys (such as Pt, Ag, Pd, Au, Pt-Pd, and Pt-Au) have excellent electrochemical catalytic oxidation activity, which has been proved to be used for the electrocatalytic oxidation of glucose [5–8]. However, due to the scarcity and high cost of these precious metals, the surface of precious metal based materials is usually easily polluted by adsorbed intermediates and chloride ions, which greatly affects the stability and sensitivity of the sensor [9, 10]. In view of this, researchers try to develop electrode materials with high performance and low cost for nonenzymatic glucose sensing. In particular, transition metal oxides have the advantages of low price and high conductivity. They are regarded as the ideal electrode active materials for nonenzymatic glucose sensing [11, 12]. Among them, Co_3_O_4_ is an ionic semiconductor with both polar positive electrodes (two Co^2+^, two Co^3+^, and four O^2-^) and polar negative electrodes (two Co^3+^ and four O^2-^). It has excellent electrochemical performance and has been widely used in photocatalysis, supercapacitors, lithium-ion batteries, electrochemical sensors, and other fields [13]. Therefore, Co_3_O_4_, which has good lasting stability and electrocatalytic activity in alkaline medium, is also one of the most promising materials for electrocatalytic oxidation of glucose.

As we all know, different morphologies and microstructures of materials would produce substantial differences in their surface area, particle size, pore structure, mass transfer, and electron transfer efficiency, which will affect their electrochemical sensing performance [14]. Therefore, construction of Co_3_O_4_ with excellent microstructure can effectively enhance the electrocatalytic performance of glucose. If the Co_3_O_4_ catalytic material is directly grown on the conductive substrate in the form of well-arranged nanoarrays, the performance of the catalytic material can be effectively improved. In this work, one-step hydrothermal method was used to prepare porous Co_3_O_4_ nanoneedle arrays (Co_3_O_4_ NNs/NF) in situ on Ni foam. With the help of the three electrode system, the electrochemical performance of the self-supporting electrode in situ was tested. The results show that Co_3_O_4_ NNs/NF exhibits higher sensitivity, lower detection limit, good repeatability, and good excellent selectivity for common interfering substances.

## 2. Materials and Methods

### 2.1. Preparation of Co_3_O_4_ NNs/NF

*Pretreatment of Ni Foam:* firstly, an area of 2 × 4 cm^2^ Ni foam was sonicated in the HCl solution (2 M), anhydrous ethanol, deionized water for 15 min, respectively, and then, the cleaned Ni foam was dried at 60°C.

*Preparation of Co_3_O_4_ NNs/NF:* 5 mmol of Co(NO_3_)_2_·6H_2_O and 4.5 mmol of urea were solved into 30 mL of deionized water. After stirring, 2 mmol of cetyltrimethyl ammonium bromide (CTAB) was added into the above solution and stirred at 45°C for 30 min. Subsequently, the uniform solution was transferred into the Teflon-sealed autoclave, and the cleaned Ni foam was inserted into the inner container by tweezers, and the Ni foam was completely immersed in the solution. Then the autoclave was sealed and placed in the electric hot air drying oven, and then heated continuously for 6 h at 120°C. When the autoclave naturally cooled to room temperature, the autoclave was opened, and the Ni foam with precursor was collected by tweezers and washed repeatedly with ethanol and distilled water. Then, the Ni foam was put it into a drying oven with a temperature set at 60°C for 8 h. Finally, the Ni foam with precursor was placed in a clean crucible and then baked in a muffle furnace. The heating rate was set at 1°C/min, heated to 350°C, and continuously calcined 2 h.

### 2.2. Electrochemical Performance Test

In current work, we prepared the sensing material on the surface of Ni foam. The thickness of sensing film is about 0.1 mm. During the electrochemical test, the RST-5000F electrochemical workstation was used for electrochemical test. The freshly prepared NaOH (0.1 M) solution was served as the electrolyte. Cyclic voltammetry and chronoamperometry were performed at room temperature. Co_3_O_4_ NNs/NF (1 × 2 cm^2^), Ag/AgCl electrode, and Pt sheet electrode were used as working electrode, reference electrode, and counter electrode, respectively. The humidity in current work is 30 RH%.

## 3. Results and Discussion

The prepared sample was obtained from the Ni foam by ultrasonic wave, and the composition of the sample was studied by XRD. The XRD pattern of Co_3_O_4_ arrays on Ni foam is shown in Figure 1. The obvious diffraction peaks at 19.0°, 31.2°, 36.8°, 38.5°, 44.8°, 55.6°, 59.3°, and 65.2° are corresponding to (111), (220), (311), (222), (400), (422), (511), and (440) planes of cubic phase Co_3_O_4_ (JCPDS No. 42-1467). Moreover, no other impurity peaks are found in the pattern, which indicates that the as-prepared Co_3_O_4_ sample has good crystallinity and high purity.

Figure 2(a) displays the SEM image of Co_3_O_4_ NNs/NF electrode at low magnification. It can be seen that Co_3_O_4_ nanoneedles are evenly covered on the conductive substrate, and there is a gap between the nanoneedles, which is conducive to the diffusion of electrolyte and the escape of bubbles on the electrode surface, so as to improve the catalytic activity. From the high magnified SEM image in Figure 2(b), it can be found that the diameter of Co_3_O_4_ nanoneedles is about 80-100 nm, and its surface is rough and uneven, which may be porous structure. Subsequently, Co_3_O_4_ nanoneedles were dispersed in ethanol by ultrasonic method and characterized by TEM technique.  Figure 2(c) shows that the nanoneedles with a diameter of about 100 nm are actually composed of interconnected single nanoparticles, which is consistent with the SEM observation. Such highly porous nanoneedle structure is helpful for the rapid diffusion of electrolyte ions in the electrode and accelerates electron transfer, so that the as-prepared Co_3_O_4_ electrode may have good electrochemical performance. Additionally, the HR-TEM image of Co_3_O_4_ nanoneedles (Figure 2(d)) shows that there are two groups of clear lattice fringes. It is found that their fringe spacing is 0.242 nm and 0.465 nm, respectively, which exactly corresponds to the (311) and (111) crystal planes of Co_3_O_4_ standard diffraction spectrum (JCPDS 42-1467). These results further confirm the successful synthesis of porous Co_3_O_4_ nanoneedles on Ni foam.

Using a typical three electrode system, the electrocatalytic activity of Co_3_O_4_ NNs/NF for glucose oxidation was investigated by cyclic voltammetry.  Figure 3(a) shows the CV curve of Co_3_O_4_ NNs/NF in the absence and presence of 0.6 mM glucose at a scanning speed of 10 mV s^−1^. Obviously, the oxidation peak current of Co_3_O_4_ NNs/NF at 0.55 V increases significantly after the addition of 0.6 mM glucose. In addition, Figure 3(b) shows the CV curve of Co_3_O_4_ NNs/NF when the glucose concentration in 0.1 M, the NaOH solution is 0 mM, 0.2 mM, 0.4 mM, and 0.6 mM, respectively (the scanning speed is set to 10 mV s^−1^). With the increase of glucose concentration, the peak current also increases. The above results show that the prepared Co_3_O_4_ NNs/NF has good electrocatalytic activity for glucose oxidation, and the specific process can be described as [15, 16]

(1) $$\begin{array}{c} {\text{Co}}_{3}{\text{O}}_{4}+{\text{OH}}^{-}+{\text{H}}_{2}\text{O}⟶3\text{CoOOH}+{\text{e}}^{-}, \end{array}$$

(2) $$\begin{array}{c} \text{CoOOH}+{\text{OH}}^{-}⟶{\text{CoO}}_{2}+{\text{H}}_{2}\text{O}+{\text{e}}^{-}, \end{array}$$

(3) $$\begin{array}{c} 2\text{Co}{\text{O}}_{2}+\text{glucose}⟶2\text{CoOOH}+\text{gluconolactone}. \end{array}$$

Figure 3(c) shows the CV curve of Co_3_O_4_ NNs/NF electrode at different scanning rates (5-50 mV s^−1^) in the presence of 0.8 mM glucose in 0.1 M NaOH. The peak current of anode and cathode increases with the increase of scanning rate. It can be seen from Figure 3(d) that the peak current of anode and cathode has a good linear relationship with the square root of scanning rate, and the correlation coefficients are 0.99381 and 0.99893, respectively, indicating that the oxidation process of glucose on Co_3_O_4_ NNs/NF is a diffusion controlled process [17].

Chronoamperometry technology was carried out to evaluate the sensitivity, detection limit, and selectivity of the electrode to glucose. Under the condition of working voltage of 0.55 V, Co_3_O_4_ NNs/NF electrode was tested, and glucose solutions with different concentrations were gradually added to 0.1 M NaOH solution. As shown in Figure 4(a), when glucose of different concentrations is added to the alkaline solution in the state of uniform stirring at an interval of 50 s, it can be seen that the current response is relatively rapid and the curve is similar to a ladder. In addition, Figure 4(b) shows the corresponding relationship between glucose concentration and current in this process. In the range of 1 *μ*M-0.338 mM, the concentration and current have good linear correlation. Its linear regression equation can be expressed as *I* (mA) = 9.14C (mM) + 0.097 (*R*^2^ = 0.99017), and the sensitivity is 4570 *μ*A mM^−1^ cm^−2^. The detection limit (LOD) for glucose is about 0.91 *μ*M (*S*/*N* = 3), and its response time is about 8 s (Figure 4(c)).

Since there are other interfering substances in real human serum, which may also be oxidized, it is necessary to test the anti-interference ability of Co_3_O_4_ NNs/NF electrode. Here, the typical disruptors were selected, such as uric acid (UA), ascorbic acid (AA), fructose, and sucrose for electrochemical detection by chronoamperometry. Because the concentration of blood glucose in normal human serum is 30-50 times that of these interfering substances [18], 1.0 mM glucose and 0.1 mM interfering substances were added for testing. It can be seen from Figure 4(d) that the current density increases significantly after adding 1.0 mM glucose, but there is no significant change in current density after adding other interferents. Therefore, Co_3_O_4_ NNs/NF has good selectivity for glucose detection.

Repeatability and stability are also important indicators to evaluate the operability and durability of the prepared nonenzymatic glucose sensor electrode. Five Co_3_O_4_ NNs/NF electrodes were prepared by the same method, and the prepared electrodes were tested by cyclic voltammetry under the same conditions. Their respective peak oxidation currents were recorded. As shown in Figure 4(e), its relative standard deviation (RSD) is 7.1%, which has good repeatability. In order to study the stability of the electrode, the Co_3_O_4_ NNs/NF electrode was placed at room temperature for 28 days, and the cyclic voltammetry test was carried out every 7 days. The oxidation current of the electrode maintains 87.1% of its initial value on the 28th day (Figure 4(f)), indicating good stability of the Co_3_O_4_ NNs/NF electrode. It can be attributed to that the active material is evenly and firmly grown on the conductive Ni foam, leading to the stable structure. It is not easy to collapse or agglomeration, so it has good repeatability and stability.

## 4. Conclusions

In this work, a simple one-step hydrothermal synthesis method of Co_3_O_4_ NNs/NF is proposed for the detection of nonenzymatic glucose. The sensor based on Co_3_O_4_ NNs/NF has good sensitivity to glucose (4570 *μ*A mM^−1^ cm^−2^) and low detection limit (0.91 *μ*M). The linear detection range is 1 *μ*M-0.337 mM. Moreover, it has good selectivity and stability for glucose. At the 28th day, its oxidation response current still maintains 87.1% of its initial value. The good electrochemical sensing performance of Co_3_O_4_ NNs/NF based sensor for glucose can be attributed to the following factors: on the one hand, the firm and evenly arranged Co_3_O_4_ nanoneedles grown directly on the conductive substrate can prevent the blockage of active sites caused by additional adhesives, so as to ensure efficient electron transfer. On the other hand, the ordered and interconnected porous structure and large specific surface area can not only provide more active sites for electrochemical reactions but also enhance the contact between active substances.

## Figures and Tables

**Figure 1:** XRD pattern of Co_3_O_4_ NNs.

**Figure 2:** SEM images of Co_3_O_4_ NNs/NF at (a) low magnification and (b) high magnification. (c) TEM and (d) HR-TEM images of Co_3_O_4_ NNs.

**Figure 3:** CV curves of Co_3_O_4_ NNs/NF (a) with and without glucose, (b) at different glucose concentration, (c) at different scan rates, and (d) the corresponding linear relationship between the anodic/cathodic peak currents and the square root of scanning rate (v^1/2^).

**Figure 4:** (a) The amperometric response of Co_3_O_4_ NNs/NF when glucose was continuously injected into 0.1 M NaOH solution at 0.55 V; the inset showed the enlarged response curve from the black rectangle. (b) Calibration curve between current response and glucose concentration. (c) The response time of Co_3_O_4_ NNs/NF. (d) The amperometric response of Co_3_O_4_ NNs/NF to the sequential addition of 1 mM glucose and 0.1 mM different interferents (UA, AA, fructose, and sucrose); Potential: 0.55 V. (e) The peak oxidation currents of Co_3_O_4_ NNs/NF fabricated in five batches via the same method. (f) Storage stability of Co_3_O_4_ NNs/NF tested by CV.

## Data Availability

The data used to support the findings of this study are available from the corresponding author upon request.
